The article "Public restrooms, periods, and people experiencing homelessness: An assessment of public toilets in high needs areas of Manhattan, New York" was published in 2021. Journal: PLoS One.

# Public restrooms, periods, and people experiencing homelessness: An assessment of public toilets in high needs areas of Manhattan, New York

**DOI:** 10.1371/journal.pone.0252946

**Published:** 2021-06-23

**Authors:** Andrew R. Maroko, Kim Hopper, Caitlin Gruer, Maayan Jaffe, Erica Zhen, Marni Sommer

**Affiliations:** 1 Department of Environmental, Occupational, and Geospatial Health Sciences, Graduate School of Public Health and Health Policy, City University of New York, New York, NY, United States of America; 2 Department of Sociomedical Sciences, Mailman School of Public Health, Columbia University, New York, NY, United States of America; Centre for Addiction and Mental Health, CANADA

## Abstract

Access to safe, clean water and sanitation is globally recognized as essential for public health. Public toilets should be accessible to all members of a society, without social or physical barriers preventing usage. A public toilet facility’s design and upkeep should offer privacy and safety, ensure cleanliness, provide required sanitation-related resources, and be gender equitable, including enabling comfortable and safe management of menstruation. Menstrual hygiene management (MHM) refers to the need to ensure that girls, women and all people who menstruate have access to clean menstrual products, privacy to change the materials as often as needed, soap and water for washing the body as required, and access to facilities to dispose of used materials. Challenges around menstruation faced by people experiencing homelessness, which tend to be greater than those facing the general population, include inadequate toilet and bathing facilities, affordability issues around menstrual products, and menstrual stigma. Public toilets are a vital resource for managing menstruation, particularly for vulnerable populations without reliable access to private, safe, and clean spaces and menstrual products. This mixed-methods study sought to: 1) understand the lived experiences of MHM among people experiencing homelessness in New York City with respect to public toilets; 2) describe general and MHM-related characteristics of public toilets in high need areas of Manhattan and analyze their interrelationships; and 3) examine the associations among neighborhood-level demographics and the public toilet characteristics in those areas. Qualitative methods included key informant interviews (n = 15) and in-depth interviews (n = 22) with people with experience living on the street or in shelters, which were analyzed using Malterud’s ‘systematic text condensation’ for thematic cross-case analysis. Quantitative methods included audits and analyses of public toilet facilities (n = 25) using traditional statistics (e.g., Spearman’s correlations) and spatial analyses (e.g., proximity buffers). Qualitative findings suggest cleanliness, access to restrooms, and availability of resources are critical issues for the participants or prospective users. Quantitative analyses revealed insufficiently provided, maintained, and resourced public toilets for managing menstruation in high-needs areas. Findings also suggest that toilets with more MHM-related resource availability, such as menstrual products and toilet stall disposal bins, were more difficult to access. Neighborhood-level characteristics showed a potential environmental injustice, as areas characterized by higher socioeconomic status are associated with more access to MHM-specific resources in public restrooms, as well as better overall quality.

## Introduction

Access to safe, clean water and sanitation is globally recognized as essential for public health [1–3]. In the United States (US) and beyond, readily accessible public toilets are considered modern necessities (even if often ill-provided [4]), important for accommodating an extremely mobile population, and particularly critical for those with greater needs such as children, the elderly, those with medical conditions requiring increased toilet use, people who are menstruating, and those experiencing homelessness [5]. Fundamental components of a public toilet include its design, its maintenance, and its accessibility; meaning, for example, a toilet should be accessible to members of the public, without social or physical barriers preventing usage, its design should provide privacy and safety, and its upkeep should ensure cleanliness [6, 7]. Additional modifications may be mandated, such as handrails for those with special needs, or as will be discussed in this paper, aspects that enable comfortable and safe management of menstruation.

Menstrual hygiene management (MHM) refers to the need to ensure that girls, women, and all people who menstruate have access to clean menstrual products, privacy to change the materials as often as needed, facilities for disposing of used materials, and soap and water for washing bodies as required [8]. There is a growing global recognition that public toilets and bathing facilities should provide these fundamentals of MHM [9, 10]. Other aspects, such as hooks to hang a bag, adequate lighting, a mirror to check for leaks, and toilet paper or paper towels can further improve these experiences [10]. Absence of adequate enabling factors for MHM contributes to anxiety, embarrassment, and shame for those who menstruate, especially given ongoing menstrual stigma and taboos [11, 12]. This hinders the ability to participate successfully in school, work, and other aspects of daily life, and contributes to perpetuating a gender inequitable society [13–15]. As more than a quarter of the US population is estimated to currently menstruate [16], access to clean, safe toilets with water, soap, and disposal mechanisms, is essential for ensuring dignified, safe, comfortable MHM for all.

Although the US-based literature remains scarce on how people with limited resources manage their menstruation, evidence from a few studies suggests that the cost of menstrual products presents particular challenges [17–19]. One survey conducted with low-income women in St. Louis, Missouri, including some experiencing homelessness, found that nearly 50% had been forced to choose between buying food and menstrual products in the last year. Many of the women, especially those experiencing homelessness, had no place to change their menstrual products, particularly at night when they felt that public toilets were not safe [18]. While documentation of the challenges around menstruation faced by people experiencing homelessness are more prevalent in the US media than in the peer reviewed literature, there is an emerging evidence base describing inadequate toilet and bathing facilities for those who live on the street and in shelters, affordability issues around menstrual products, and experienced menstrual stigma [17, 19, 20].

Homelessness represents a long-standing public health crisis in the US in general, and New York City (NYC) specifically. In September 2019, there were over 62,000 people in NYC’s shelter system each night; a number that does not account for the many additional unhoused people living with friends, family, or on the street [21]. A point-in-time count assessment estimated that there were over 3,500 individuals living on the street in January 2019, a number likely to be an underestimation [22]. In addition, the shelter system served over 133,000 separate individuals in 2018, a 59% increase over the prior decade [21]. Access to basic resources is among the many challenges facing this population, including safe and stable shelter, proper nutrition, health care, and toilet facilities. The COVID-19 pandemic has only served to exacerbate these challenges.

Public toilets, or restrooms as they are frequently called, are a vital, but often overlooked, resource for MHM, particularly for vulnerable populations such as those experiencing homelessness who may lack reliable access to private, safe, and clean spaces or menstrual products. Of importance to note, this includes access to public versus private toilets, particularly in large urban environments [6]. Public toilets are facilities funded by federal, state or local dollars, technically open to anyone. They range from stand-alone restrooms, such as those in parks or on street corners, to those tied to publicly accessible institutions, such as free museums, transportation systems, or libraries. Although in theory open to the public, access to such toilets may be uneven, and limited in practice by the operating hours of the institution or park in which they are located, the “informal gatekeeping” by the staff, and may range in quality (e.g., cleanliness, stocking of toilet paper) depending on how well resourced and maintained such facilities are by the responsible government entity. Private toilets in this paper refer to those owned and maintained by private sector or commercial entities such as restaurants, coffee shops, and other stores. Access to such toilets is often limited to the paying clientele of the institution, or to those who are able to “pass” as paying customers. The passing requirement frequently translates into denial of access to populations experiencing homelessness, including those who are menstruating and in need of more frequent access [23].

Access and accessibility, as will be applied in this paper to public toilets and related resources for MHM, are concepts that are often constructed from a number of related dimensions. For instance, in health care, the dimensions can be defined as: 1) affordability (e.g., does utilization of the resource result in financial burden); 2) availability (e.g. is there enough of the resource for the demand of the population); 3) accessibility (is the resource geographically accessible and is its distribution equitable); 4) accommodation (e.g., does the resource meet the constraints and preferences of the population); and 5) acceptability (e.g., is the resource appropriate and relevant to the population’s needs and cultural setting) [24, 25]. As this relates to public toilets and MHM for people experiencing homelessness, this can be thought of as “are there enough public toilets in high-needs areas?”; “do the existing public toilets supply the requisite resources?” (e.g. stocked supply of soap; menstrual product vending machines; menstrual product disposal bins or trash cans); “are there barriers to utilization of the toilets?” (e.g., security guards screening entry into institution; expectation of payment such as a subway fare; requirement to request a code or key to restroom); and “are the characteristics (e.g., cleanliness and safety) of the toilet facilities appropriate for MHM for this population and on terms acceptable to them?”

An important feature of resource access, be it to toilets or menstrual products, is equity in the spatial distribution of resources. These “spatial justice” issues can be seen in a wide range of phenomena. For instance, the environmental justice literature has exposed many instances where exposures to environmental insults (e.g., air pollution, toxic exposures) [26–29] and more general environmental “bads” (e.g., fast food outlets, vacant and derelict land) [30–35] are increased in communities with higher proportions of people of color, foreign born residents, or lower household incomes or educational attainment. Similar findings have been reported around access to environmental “goods” such as parks and open space [34–37], healthy foods [38, 39], and health services [40–42]. However, it is unclear how or if neighborhood-level demographics associate with qualities and characteristics of public toilets.

For our purposes, this is particularly important in considering how public toilet access may impact those experiencing homelessness in relation to managing menstruation. The media has showcased how many large urban areas of the US (e.g., Los Angeles, Seattle), lack adequate public toilets and are grappling with the related implications for populations living on the street [43, 44]. In NYC, a recent media inquiry explored the inadequacy of public toilets in the city’s vast subway system (some 420 stations). The reporting described toilets turned into storage closets, variable hours of service, and major challenges in maintenance and cleanliness [45]. The public at large would likely benefit from improved, safe, clean public toilets. For those living on the street or in shelters–routinely denied access to the numerous private sector toilets in restaurants, cultural institutions, cafes, and shops–the lack of clean, accessible public toilets presents distinct challenges. However, to date, little research has systematically explored access to public toilets in the US for people experiencing homelessness, especially with respect to managing their menstruation.

This study sought to: 1) better understand the lived experiences of menstrual management or MHM among people experiencing homelessness in NYC with respect to public toilets; 2) describe general and MHM-related characteristics of public toilets in high need areas of Manhattan and analyze their interrelationships; and 3) examine the associations among neighborhood-level demographics and the public toilet characteristics in those areas.

## Methods

We conducted a mixed-methods study that sought to capture, at individual, institutional, and ecological levels, the nature of menstrual management on the part of those experiencing homelessness, and how the local context may shape those experiences. This included: 1) key informant interviews with staff of government agencies and homeless service organizations; 2) in-depth interviews with people experiencing homelessness who menstruate; and 3) audits of public toilet facilities in a select number of sites across the borough of Manhattan in NYC. This paper will focus on select findings from the qualitative data, and quantitative insights gained from public toilet audit data. The qualitative information served to enhance and guide our understanding and interpretation of the toilet audit data.

### Qualitative methods

Our sample for the key informant interviews (n = 15) included staff of government agencies and organizations providing services to people experiencing homelessness, including shelters. Our sample for the in-depth interviews (n = 22) included street and sheltered individuals experiencing homelessness who were ages 18 years and older and who menstruate. We sought to identify 4–5 individuals in each of the following age groups: 18–25; 26–35; 36–45; and 46 and above in order to capture a range of menstruation-related experiences (more in-depth methods described in Sommer et.al. 2020 [23]). The participants all presented as female, although we did not ask for gender identification. Similarly, we did not probe on exact age beyond confirming they were above 18 years of age, given the sensitivity of the population. However, a number of participants offered their age during the interviews, and the researchers estimated the age of the others based on appearance and life story. Based on these methods, we can approximate that the participants ranged from ages 18–62, including 8 in the 18–25 category, 5 in the 26–35 category, 4 in the 36–45 category, and 5 in the 46 and above category. All participants provided oral consent prior to participating.

Participants were recruited during the months of June–August 2019, with recruitment ending when we reached data saturation. Key Informants were recruited through electronic outreach to organizations known to be relevant to homeless services and/or public toilets provision in NYC. The majority of key informant interviews were conducted online using free conference call, with a small number conducted in the offices of those being interviewed, depending on the preference of the key informant. Recruitment for those experiencing homelessness occurred through the Coalition for the Homeless as well as from an organization specifically serving homeless youth. Both organizations placed a flier in their lobby and made announcements about the study including an incentive ($10 or $15 metro card) to the population who they serve. Clients who expressed interest in participating in the study were introduced to the research team by the Coalition or service provider. All of the interviews conducted with the homeless population occurred in private rooms (e.g. empty offices) at the Coalition or other service provider.

Our decision to focus on Manhattan was both pragmatic and strategic. Although the shelter system is scattered throughout NYC’s five boroughs, annual street counts routinely find many more street-dwelling homeless in Manhattan than in the other boroughs of NYC (excluding subways) [46].

The study received Internal Review Board (IRB) approval from the Columbia University Medical Center (CUMC) Institutional Review Board. A waiver of written consent was requested and approved by the CUMC IRB on the basis that the only record linking the subject and the research would be the consent document and the principal risk of the study was the potential harm resulting from a breach of confidentiality. In consultation with the Coalition for the Homeless, we concluded that a written consent form may also be an issue due to varying literacy of those experiencing homelessness. A consent tracking sheet was maintained to ensure all participants’ consenting was documented.

### Public restroom audit

In order to quantify differences in public toilets, an audit instrument was created by combining and adapting existing instruments used to assess the accessibility and acceptability of toilets in global development programs in both humanitarian and development contexts [47]. These tools assess multiple elements of the toilet design including structure and hardware, availability of basic supplies, and safety and privacy features. Data collected by our customized audit instrument included basic information (e.g., location, number of toilets), cleanliness (e.g., floors, toilets, sinks), data on availability of general resources (e.g., soap, toilet paper, trash cans, hooks on the back of stall doors for hanging clothing or bags, locks on stall doors), permission and economic-based accessibility (e.g., permission needed to use toilets, purchase required, codes or keys needed, access to the establishment needed), other accessibility characteristics (e.g., hours of operation, signage, gender neutral restrooms), and availability of MHM-specific resources. The latter included availability of menstrual products such as freely accessible or vending machine-provided menstrual pads or tampons, and disposal bins, which are refuse receptacles near the toilet (e.g. trash can) or within the toilet stall (e.g. small unit on the stall wall). Such internal stall bins eliminate the need to carry a used product to a garbage receptacle situated in a public space (e.g., the shared larger restroom). It is important to note that all of the variables collected, such as hooks on doors and privacy assured by locks on stall doors, are relevant to enabling comfortable, safe and dignified MHM, even if they are not MHM-specific. The majority of variables are binary (yes/no), simply indicating the presence, or lack, of a certain feature or characteristic (e.g., a disposal bin). However, the cleanliness variables were coded on a 5-class Likert scale.

Prior to data collection, the full research team met to discuss the tool and reach consensus about the categories included. After the tool was developed, it was field tested, and upgrades were made to improve usability and functionality. This involved discussing the general process for auditing a public toilet facility, including minimizing disruption of usual practice, making careful observations, and performing functionality tests on the hardware (e.g., locks, sinks, hand dryers). In addition, researchers discussed the definition of each variable to ensure common understanding and consistency in utilizing the audit tool. Particular emphasis was placed on the cleanliness variables (Likert scales) as they are the most open to subjectivity. Between July 12 and September 3, 2019, researchers performed the audits in teams of two or more, with one of the researchers participating in every audit to ensure consistency in coding.

#### Spatial methods—Identifying high-needs areas of people experiencing street homelessness

Various data sources were reviewed to identify places within Manhattan which may have a higher need for public toilet facilities. These included various homelessness counts and censuses, shelter locations and capacity, and others. Ultimately, locations of “hot spots,” identified with the assistance of the Manhattan Outreach Consortium (MOC) as of April 2019, were used as they proved to be more stable and spatially discrete than other options explored (Fig 1). These are not geographic statistical hot spots (e.g., as calculated by spatial distribution statistics), but rather places where people are known to congregate or “bed down.” They are identified mainly through ongoing outreach efforts and updated monthly. It is important to note that locations may change over time due to relocation of the individuals (e.g., some people may get sheltered, accept outreach offers, be asked to disperse by the police, or move to another neighborhood). Gender breakdowns, although important, were more difficult to estimate due to a lack of reliable or complete data and thus are not included in the analysis. This “hot spot” information is used to identify potentially high-needs locations (i.e. locations with greater numbers of people experiencing homelessness) to perform the public toilet audits (see below).

**Fig 1:** “Hot spot” locations of people experiencing homelessness (April 2019). Locations are displayed with intentional locational error for privacy and safety concerns.

Public toilet audit areas were defined by creating ½ mile (~ 805 meters) radius buffers from selected hot spot / encampment locations. As many of these locations are spatially clustered, some audit areas included multiple encampments of individuals who are living on the street or “sleeping rough.” The team walked all streets and accessible park and open spaces intersecting the buffer areas and identified all publicly accessible toilets (e.g., within parks, subways, libraries, commuter train stations, public museums). It is important to note that the researchers only audited *public* restrooms, and did not assess private businesses (e.g., coffee shops, restaurants, bars) or those found in shelters or other facilities. This was because shelter facilities may be unavailable during the daytime for those staying there, and because those sleeping on the street tend not to access shelter facilities if they are not sleeping there. The data collection resulted in the identification of 31 publicly accessible toilet facilities. However, six were out of order, closed, or otherwise inaccessible resulting in 25 fully audited facilities (Fig 2).

**Fig 2:** Audited public toilet facilities in Manhattan, NY (n = 25).

### Analysis

#### Qualitative analysis

All of the qualitative data (KIIs and IDIs) was transcribed and analyzed by two of the researchers using Malterud’s ‘systematic text condensation’ for thematic cross-case analysis [23]. This included the following steps: (1) identification of preliminary themes; (2) creative development of qualitative codes; (3) condensation of coded text; (4) synthesis and reconceptualization. The PI reviewed and helped to revise the final codebook, and the analysis team used Dedoose analytic software to code the data. The key themes were shared with the full research team for discussion, refinement and validation. The section below presents the key analytical themes and supporting textual passages of relevance to the public toilet audit data insights.

#### Quantitative (audit data) analysis

Statistical analyses were performed in SPSS (IBM Corp., Armonk, NY) and spatial analyses in ArcMap 10.7 (ESRI, Redlands, CA). Collected data from the audits were explored in a number of ways. First, simple indices were created to capture broad domains of public toilet-level characteristics. Second, descriptive statistics of the indices were calculated to show the overall characteristics of the public toilets in these high-needs areas. Third, the indices were compared to one another using Spearman’s correlations. And finally, bivariate associations among public toilet characteristics and contextual neighborhood-level socioeconomic data were explored.

Simple indices were created to represent major domains of public toilet facility characteristics. These include (1) cleanliness, (2) general resource availability (availability 1—general), (3) MHM-specific resource availability (availability 2—MHM), (4) accessibility with respect to permissions or purchases (access 1—permissions), and (5) accessibility with respect to hours of operation, visibility, and inclusiveness (access 2—other). Raw data were converted into index values by summing the individual variables and then using linear transformations, so that all the resulting index scores were between 0–1. For the cleanliness index, scores were not impacted by missing features (e.g., if there was no trash can or disposal bin present the cleanliness score was not affected; however, it would be reflected in the availability score). A simple additive index was then created (full index) which represents the sum of the individual domain indices, resulting in possible values ranging from zero to five.

In order to compare public toilet facility characteristics to the broader social contexts in which they are situated, “neighborhoods” had to be defined and operationalized. Locations of audited public toilets were geocoded using ArcGIS World Geocoding Service and manually checked for accuracy. American Community Survey (ACS) 5-year estimates (2014–18) at the Census Block Group (CBG) level were acquired via IPUMS / National Historical GIS [48] and mapped to represent sociodemographic characteristics of the residential population. ACS data include total population, poverty status, per capita income, median rent, non-Hispanic (NH) White residents, NH Black residents, Latinx/Hispanic residents, and adult population who did not graduate from high school (Fig 3).

**Fig 3:** Manhattan Census Block Group demographics shown in quartiles. Top row (from left to right): per capita income, percent of the population below the federal poverty level, median rent, percent of the adult population without a high school diploma. Bottom row (from left to right): percent NH White, percent NH Black, and percent Latinx/Hispanic.

As the public toilet point locations served as the unit of analysis, pedestrian-accessible network distance buffers of 0.25 miles (~ 0.40 km) were created (Fig 4). These network buffers differ from fixed-distance (“as-the-crow-flies”) buffers as they reflect areas within a walkable distance along the network (pedestrian-accessible streets and paths). Because the buffer boundaries do not conflate with CBG boundaries, the ACS data were attributed to each public toilet by using areal weighting. This method of data disaggregation is a type of dasymetric approach, where a second dataset (in this case area), is used to reapportion the variable of interest (in this case ACS data). Areal weighting assumes a homogeneously distributed population, which although committing ecological fallacy, has been shown to provide more meaningful estimates than other, non-dasymetric, neighborhood estimation techniques (e.g., centroid containment, intersection) [49–52]. In the case of this study, CBGs intersected by the network buffer are split, creating “child” polygons. The area of each child polygon is calculated and the variable of interest (e.g., total population) is disaggregated to the new polygons by multiplying the CBG value by the ratio of the child polygon area divided by the original CBG area. For instance, if there were 1000 residents in a CBG, and the network buffer included 50% of the CBG area, it would be assumed that 500 residents (50%) lived in within the buffer area. Public toilet-specific demographic and socioeconomic contexts (“neighborhoods”) were then calculated by summing count variables in all child polygons within the public toilet’s network buffer. Non-count variables (e.g., median rent) were calculated using population-weighted means.

**Fig 4:** Quarter-mile (~0.4 km) pedestrian-accessible network buffer around one public toilet location.

## Results

### Qualitative

The qualitative findings served to reveal the human experience behind the toilet audit findings, enriching and guiding our interpretation of the audit data. As reported elsewhere [23], the most prevalent challenges that emerged from the interviews pertained to accessibility, resource, cleanliness, and safety issues. This proved to be the case both for those living on the street and those living in shelters, the latter of whom also need facilities as they move around the city when seeking out services or employment.

#### Inadequate maintenance of public toilets

Specific challenges included significant concerns around the cleanliness of many public toilets; a common refrain was wondering whether public toilets were ever used, particularly in the subway system, combined with comments about the challenges their lack of upkeep posed:

*I think I’ve used the subway bathroom like twice in my life…And it was disgusting…The smell. Mostly the smell…you notice little things in there, like the sink might be a little dirty, the tissue might be all over the floor, so, mm, it’s just nasty. I wouldn’t, if I could avoid it, I would… –IDI017*

Many informants also expressed concerns about their lack of maintenance, with recommendations emerging from the respondents that corresponded to the types of cleanliness challenges observed during the toilet audits:

*Clean the bathrooms enough to where someone can go in and make sure we have the necessities, soap, napkins, the dryer, even if there’s no dryer…Maintain [them] that way.–IDI14*

For their part, key informants based in service organizations or local government, described challenges related to the provision and maintenance of public toilets, such as resource limitations that constrain hours of operation. Parks department informants, for example, bemoaned the lack of staff needed to ensure that public toilets could be adequately cleaned in order to open on time at 8am (especially if they had been “trashed” the night before). Given the centrality of park-based toilet facilities (referred to as “comfort stations”) as a daytime resource for those needing a public toilet, uncertainty with respect to hours of operation, cleanliness and adequate supplies is a routine worry. When special effort is made to address MHM, other city employees report, vandalism can make short work of, say, menstrual product vending machines in public facilities:

*We did try sanitary napkins and tampons [in dispensers] at one point*, *but*, *people broke in and just…This was quite a while ago*, *but*, *people would*, *you know*, *try and either take the products*, *light ’em on fire*, *have fun with them*, *whatever it is that they do*, *because that is the reality*.–KII 03

The latter example highlights the challenge facing city government in the provision of more accessible and MHM-friendly public toilet facilities, particularly if there are insufficient resources for monitoring their usage and/or maintenance. However as with the maintenance issue, the homeless respondents had suggestions in relation to improving the accessibility and MHM-friendliness of facilities:

*If, you know, it were up to me, I would have bathrooms, just, a lot of bathrooms…bathrooms with locks, one stall, privacy, um. I honestly wouldn’t even mind if the, I don’t know what it’s called but there were machines, you paid a quarter, I wouldn’t mind if we went back to the twenty-five cent tampons, just I wish there were access, cause I don’t carry pads if I don’t expect my period….but I feel like just the event of getting your period is such a mission, to like put on a pad, it’s like, there should be a bathroom 5, 10 minutes away, with access to stuff like that for free, hopefully one day.–IDI13*

#### Inadequate hours of operation

Informants also complained about the limited numbers of public toilets throughout the city, and their restricted hours of operation, such as those located in the city’s parks. As one respondent shared:

*So, you have to, like, go to the subway to use the bathroom, and those are closed from midnight to 5am. They’re, um, they don’t even always open them at 5am.–IP2*

As many noted, periods do not stop flowing at nighttime, yet public toilets become almost inaccessible. As another informant suggested, the restriction of hours–similarly found in the toilet audit data–was potentially purposeful:

*They just don’t want people in it, because they know that that’s the place where homeless people go…like, you know, um, so they know that at a certain time at night, if they close it, that this is only when homeless people are going to be in there. _IDI003*

### Toilet audits

Such cautionary statements provide a sound prelude to our own inspections. In reviewing the basic descriptive information about the audited public toilets (n = 25) and their respective neighborhoods, there emerged a fair amount of variation in most of the variables (Table 1). For instance, although all of the audited public toilets had running water and adequate lighting available, not all had functioning stall doors and locks (96% and 92%, respectively). Additionally, only 60% (n = 15) provided hooks or shelves for bags, clothing or belongings (a component of the general resource availability index, and useful for those carrying menstrual products with them). Cleanliness scores also demonstrated a wide range of values with all variables ranging between 1 (least clean) to 5 (most clean).

**Table 1:** Variables associated with audited restrooms.

Category	Variable	Variable Type	Min.	Max.	Criteria Met (%)^a^	Mean^b^	Std. Dev.^b^
Cleanliness^c^	Floors	Likert	1	5	N/A	3.56	1.23
	Toilets	Likert	1	5	N/A	3.64	1.22
	Sinks	Likert	1	5	N/A	3.80	1.19
	Trash Cans	Likert	1	5	N/A	4.39	1.16
	Disposal Bins	Likert	1	5	N/A	4.25	1.39
Availability -1 General Resources	Soap	Dichotomous	0	1	76	N/A	N/A
	Hooks	Dichotomous	0	1	60	N/A	N/A
	Water	Dichotomous	1	1	100	N/A	N/A
	Functional Toilet Seats	Dichotomous	0	1	96	N/A	N/A
	Functional Stall Door	Dichotomous	0	1	96	N/A	N/A
	Functional Lock	Dichotomous	0	1	92	N/A	N/A
	Adequate Light	Dichotomous	1	1	100	N/A	N/A
	Toilet Paper	Dichotomous	0	1	88	N/A	N/A
	Paper Towels	Dichotomous	0	1	44	N/A	N/A
	Hand Dryer	Dichotomous	0	1	88	N/A	N/A
	Trash Cans	Dichotomous	0	1	88	N/A	N/A
	Mirror	Dichotomous	0	1	68	N/A	N/A
Availability -2 MHM Resources	Disposal Bins	Dichotomous	0	1	24	N/A	N/A
	MHM Vending Machine	Dichotomous	0	1	12	N/A	N/A
	Free MHM Products	Dichotomous	0	0	0	N/A	N/A
Access– 1 Permissions	Permission not needed to use toilets	Dichotomous	0	1	92	N/A	N/A
	Purchase not needed to access toilets	Dichotomous	0	1	96	N/A	N/A
	Code or key not needed	Dichotomous	1	1	100	N/A	N/A
	Access to establishment is not needed	Dichotomous	0	1	24	N/A	N/A
Access– 2 Other	Open 24/7	Dichotomous	0	1	16	N/A	N/A
	Visible Signage	Dichotomous	0	1	88	N/A	N/A
	Gender Neutral	Dichotomous	0	1	16	N/A	N/A
Indices^d^	Cleanliness	Continuous	0.06	1.00	N/A	0.71	0.26
	Availability-1 (general)	Continuous	0.42	1.00	N/A	0.83	0.16
	Availability-2 (MHM)	Continuous	0.00	0.67	N/A	0.12	0.19
	Access-1 (permissions)	Continuous	0.50	1.00	N/A	0.78	0.15
	Access-2 (other)	Continuous	0.00	1.00	N/A	0.40	0.22
	Full Index	Continuous	1.81	3.75	N/A	2.96	0.52
Neighborhood Demographics (network buffer)	Population	Continuous	2,743	16,233	N/A	8,884	3,858
	Per Capita Income ($)	Continuous	17,519	182,662	N/A	67,039	44,684
	% in Poverty	Continuous	6.3	40.7	N/A	19.7	9.9
	Median Rent ($)	Continuous	998	3,023	N/A	1,763	711
	% w/o High School	Continuous	0.6	44.8	N/A	14.6	12.7
	% NH White	Continuous	4.8	80.9	N/A	41.2	28.2
	% NH Black	Continuous	0.0	68.5	N/A	18.9	24.7
	% Latinx	Continuous	4.6	89.0	N/A	25.8	23.6

^a^ “Criteria Met” represent the proportion of restrooms which meet the variable criteria (e.g., presence of a disposal bin) is only presented for dichotomous variables. “True” is coded as 1 and “false” is coded as 0.

^b^ Mean and standard deviations are only presented for ordinal or continuous variables.

^c^ Cleanliness variables were collected as Likert scales (1–5) where “1” is least clean and “5” is most clean.

^d^ Index values are continuous and have possible ranges from 0–1 other than the Full Index which has a possible range from 0–5.

With respect to MHM-specific resources, only 24% of restrooms (n = 6) had disposal bins within stalls, 12% (n = 3) had menstrual product vending machines, and none provided free products. Overall, 17 of the 25 (68%) restrooms had no MHM-specific resources at all. Of the three MHM-specific resources (disposal bins, free products, vending machines), only one public toilet had both disposal bins and a vending machine. Of the eight which had any sort of resource, two were in parks (vending machines), two in transit stations, and the remainder were housed within various institutions (e.g., museum, department of motor vehicles, NYC job center).

Access data shows that most of the public toilets themselves did not require specific permissions or purchases, with 92% not requiring permission to use the toilet (e.g., asking an officer in the police station to use the restroom) and 96% did not require a purchase to access the toilets (e.g., needing special access to enter the establishment such as a subway station where the fare must first be paid to get to the area where the toilet is located). None required a key or electronic access code, in contrast to what individuals may encounter in some commercial establishments. However, over 75% of the restrooms required researchers to first enter or gain access to the establishment (e.g. museum, library, some park facilities or transit stations—which may not require payment but may be experienced differently based on one’s ability to “pass”). Additionally, only four (16%) were open continuously (24 hours per day, 7 days per week), all of which were either inside a police station or major transit hub. Note that even continuously open restrooms may not, in practice, be continuously available (e.g., long periods of closure for cleaning or maintenance).

Characteristics of the residential populations living around the audited public toilets (“neighborhood” variables) showed wide variation. There were large differences in all measured indicators for income (e.g., population-weighted mean per capita income ranged from approximately $17,500 to over $182,000; poverty rates from 6% to 41%), educational attainment (e.g., rates of adults without a high school degree from less than 1% to nearly 45%), and race/ethnicity (e.g., proportion of NH white populations from under 5% to over 80%).

Bivariate two-tailed Spearman’s correlations show the associations among restroom indices (Table 2). These data suggest that permissions and purchase-related accessibility (Access-1) is inversely related to the availability of MHM-specific resources (Availability-2; -0.588, p = 0.002)–*meaning the more accessible a restroom is*, *the less likely it is to have these resources*. Other associations show that cleanliness is positively associated with the availability of general resources (0.685, p < .001). This suggests that cleaner restrooms tend to have more general resources, which may be a function of more frequent maintenance and upkeep.

**Table 2:** Spearman’s correlations of restroom indices.

	_Cleanliness_		Availability-1		Availability-2		Access-1		Access-2	
			_(general)_		_(MHM)_		_(permissions)_		_(other)_	
	Rho	*(p)*	Rho	*(p)*	Rho	*(p)*	Rho	*(p)*	Rho	*(p)*
Cleanliness	--	--	0.685	*(<0*.*001)*	0.125	*(0*.*551)*	-0.055	*(0*.*792)*	-0.010	*(0*.*961)*
Availability-1 (general)	0.685	*(<0*.*001)*	--	--	0.319	*(0*.*120)*	-0.121	*(0*.*566)*	0.198	*(0*.*342)*
Availability-2 (MHM)	0.125	*(0*.*551)*	0.319	*(0*.*120)*	--	--	-0.588	*(0*.*002)*	0.306	*(0*.*137)*
Access-1 (permissions)	-0.055	*(0*.*792)*	-0.121	*(0*.*566)*	-0.588	*(0*.*002)*	--	--	-0.181	*(0*.*386)*
Access-2 (other)	-0.010	*(0*.*961)*	0.198	*(0*.*342)*	0.306	*(0*.*137)*	-0.181	*(0*.*386)*	--	--

Two-tailed Spearman’s correlations were also calculated to assess the associations among restroom index values and neighborhood demographics (Table 3). Higher indicators for income and wealth tended to correspond with more availability of resources as well as overall public toilet facility quality. For instance, higher median rents were positively correlated with more availability of general resources (0.372, p = .067), MHM resources (0.506, p = 0.010), “other” access (0.367, p = 0.071), and the full index (0.445, p = 0.026). Per capita income showed a similar trend; however, only availability of MHM resources had a meaningfully low p-value (0.408, p = .043). The proportion of the population below the federal poverty level and adults without high school degrees both showed negative correlations with MHM resource availability (-0.408, p = .043 and 0.397, p = 0.050, respectively) and the full index (-0.432, p = 0.031 and -0.381, p = 0.061, respectively). With respect to race and ethnicity, higher proportions of NH White populations were associated with greater general availability (0.349, p = 0.087) and NH Black populations with fewer permission or purchase-related access obstacles (0.360, p = .077). However, higher proportions of NH Black populations were also negatively associated with restroom cleanliness (-0.396, p = .050), general resource availability (-0.596, p = .002), and the full index (-0.538, p = .006). The only racial/ethnic variable which showed an association with MHM resource availability was a negative correlation with proportion of the population who are Latinx (-0.362, p = 0.075).

**Table 3:** Spearman’s correlations of restroom indices and neighborhood demographics.

	_Cleanliness_		Availability-1 _(general)_		Availability-2 _(MHM)_		Access-1 _(permissions)_		Access-2 _(other)_		_Full Index_	
	Rho	*(p)*	Rho	*(p)*	Rho	*(p)*	Rho	*(p)*	Rho	*(p)*	Rho	*(p)*
Per Capita Income	0.120	*(0*.*567)*	0.200	*(0*.*337)*	0.408	*(0*.*043)*	-0.119	*(0*.*570)*	0.140	*(0*.*504)*	0.292	*(0*.*157)*
% in Poverty	-0.245	*(0*.*238)*	-0.283	*(0*.*170)*	-0.408	*(0*.*043)*	0.128	*(0*.*540)*	-0.247	*(0*.*234)*	-0.432	*(0*.*031)*
Median Rent	0.234	*(0*.*260)*	0.372	*(0*.*067)*	0.506	*(0*.*010)*	-0.186	*(0*.*374)*	0.367	*(0*.*071)*	0.445	*(0*.*026)*
% w/o High School Degree	-0.196	*(0*.*349)*	-0.208	*(0*.*318)*	-0.397	*(0*.*050)*	-0.017	*(0*.*935)*	-0.200	*(0*.*338)*	-0.381	*(0*.*061)*
% NH White	0.203	*(0*.*331)*	0.349	*(0*.*087)*	0.242	*(0*.*245)*	-0.118	*(0*.*576)*	0.226	*(0*.*277)*	0.368	*(0*.*070)*
% NH Black	-0.396	*(0*.*050)*	-0.596	*(0*.*002)*	-0.317	*(0*.*122)*	0.360	*(0*.*077)*	-0.328	*(0*.*109)*	-0.538	*(0*.*006)*
% Latinx	-0.036	*(0*.*864)*	-0.071	*(0*.*735)*	-0.362	*(0*.*075)*	-0.108	*(0*.*607)*	0.009	*(0*.*965)*	-0.211	*(0*.*312)*

## Discussion

This study offers independent support of MHM difficulties previously reported for New Yorkers experiencing homelessness. Specifically, it shows that likely high need areas of Manhattan, those hosting concentrations of people experiencing homelessness, are also wanting in resources for adequate MHM. Qualitative interviews suggest that public toilet-based access to MHM products and resources (e.g. products, disposal bins) is a pressing concern for people experiencing homelessness. Our quantitative results support such worries; none of the toilets audited in our sample provided free products, and nearly 70% had no MHM-specific resources at all. Given the likely higher reliance on public toilet facilities by people experiencing homelessness, this paucity of resources, described as basic and fundamental needs for people who menstruate, almost certainly has a differential effect based on socio-economic status and unequal access to non-public alternatives.

The above inequity is further exacerbated by the quantitative findings which suggest that public toilets with more MHM-related resource availability tended to be more difficult to access with respect to needed permissions or purchases, which is in turn compounded by the fact that the vast majority (84%) of audited public toilets are not open overnight. The qualitative interviews revealed the latter to be an important barrier to menstrual management.

Pointedly, too, access to public toilets may include hidden costs or location-specific permissions–whether economic (e.g., pay for subway access) or social (e.g., ask an attendant at a museum). Negotiating these is often further complicated for people experiencing homelessness by the need to present themselves convincingly as otherwise: to “pass” as not homeless. Elsewhere, we have shown how access to private toilets, those located within private sector or commercial entities, is encumbered by this symbolic requirement [23]; public toilets, too, often come laden with their own de facto gatekeepers.

There were also detectable differences in neighborhood-level characteristics based on public toilet qualities. For instance, the public toilet facilities which provided any sort of MHM resources were positively associated with higher income and higher rent areas—and negatively associated with higher proportions of Latinx residents, lower educational attainment, and people living in poverty. Put simply, MHM resources in public toilet facilities were more prevalent in areas characterized by high socioeconomic status, as opposed to areas which may already be under-resourced or marginalized, and as such benefit more from their availability and accessibility. Overall public toilet quality followed the same trend, indicating that neighborhoods which have higher shares of vulnerable residents tend to have lower quality public toilet facilities with fewer MHM resources. This is particularly true for neighborhoods with high proportions of NH Black residents, where the toilets tended to be less clean, have less availability of general resources, and have lower overall quality. These issues may be associated with maintenance and upkeep and were revealed as important aspects of MHM based on qualitative interviews.

It is important to be reminded that the overall quality of the public toilet facilities (which included variables describing cleanliness, privacy, safety, and accessibility), *are essential for*, even if not specific to, MHM. This suggests an environmental injustice, where neighborhoods have differential access to “environmental goods” based on the sociodemographic nature of the residents. As the public toilet facilities that were audited were associated with clusters of people experiencing homelessness who may be menstruating, this has significant implications for their access to private, hygienic spaces for managing their menstruation safely and comfortably as needed. Although a preferential solution would be housing for all, and so reduce the unmet need that public toilet facilities in urban areas are expected to address, the exigency of menstrual management is one that lasts day and all night during a given menstrual period. Hence, safe access to clean public toilets is essential for anyone, housed or otherwise, moving about the streets of Manhattan. If anything, the COVID-19 pandemic has intensified such concerns, and made contagion the metric of solidarity.

It is important to note the limitations of this study. First, there were a small number of samples (25 audited public toilets, only audited once each) which may result in unstable statistical findings and would benefit from a more complete (e.g., 100%) sample of the borough. Second, the areas of Manhattan selected for auditing were based on data which are not necessarily representative of the true distribution of people experiencing homelessness, but rather rely on locations identified by homelessness outreach workers as “hot spots” at a specific point in time. Nor were we able to identify any potential bias in the spatial distribution of women or other people who menstruate who would benefit most from MHM resources. Third, this data uncertainty is linked to the inability to perform a true supply-and-demand type of analysis. As such, this study does not examine a central aspect of accessibility or availability in terms of “amount per person,” but rather just the *qualities* of the amenities that exist. It may be argued that any public toilet is better than no public toilets; however, based on the interviews, many women that are experiencing homelessness avoid public toilets specifically *because* they are not seen as clean, safe, or hygienic. Although the study design and data did not allow for a supply-demand analysis, there was large variability in the number of public toilets, and more so in the number of individual toilets/stalls within those facilities, in any given audited area. For instance, some downtown locations (e.g., near Stuyvesant Town and parts of the East Village) had no nearby public toilet facilities. Conversely, audited locations near major transit hubs or regional attractions often had over 20 individual toilets/stalls in nearby public toilet facilities.

## Conclusion

Overall, interviews suggest that public toilet facilities in Manhattan simply do not meet the menstrual hygiene management needs of women experiencing homelessness in terms of accessibility, cleanliness, privacy, or resource provision. The spatial distribution of higher and lower quality public toilet facilities, reinforced by, and interpreted through, the findings from qualitative interviews, may be an example of an environmental or spatial injustice in neighborhoods proximal to “hot spots” of people experiencing homelessness in Manhattan. Such mixed-methodological approaches are a useful way to identify and highlight such inequities; insights that may have been incomplete without the convergence of findings. The overall lack of menstrual hygiene resources in all public toilets is further exacerbated by the findings that these resources tend to be found more often in public toilet facilities which are difficult to access. Ultimately, we believe that if these spatial biases, accessibility and resource issues, and overall paucity and poor quality of supply are addressed in Manhattan, it would not only contribute to meeting the needs of the most marginalized or vulnerable populations (e.g., people experiencing homelessness), but provide substantial benefits for the public good. That such needs are exacerbated during the global COVID-19 pandemic adds ever more urgency.
